This article has been retracted.

# The Application of DOMS Mechanism and Prevention in Physical Education and Training

**DOI:** 10.1155/2022/9654919

**Published:** 2022-01-07

**Authors:** Cong Zeng, Ge Luo, Shijun Xu, Yi Li

**Affiliations:** ^1^Sports Department, Liuzhou Institute of Technology, Liuzhou 545616, China; ^2^Physical Education College, Guangxi University of Science and Technology, Liuzhou 545006, China; ^3^Sports Department, Guangxi Medical University, Nanning 530021, China

## Abstract

To analyze the causes of muscle soreness and injury during precompetition training in university sports meet and taking the DOMS mechanism as the main line to find a reasonable way to deal with the muscle pain and prevent the injury, 125 college students participating in stadium games training were randomly selected. The muscle pain and injury during the training were obtained through interviews, mathematical statistics, and literature review. The information of exercise load, pain and injury type, exercise ability, pain degree, and recovery time was comprehensively analyzed to study the mechanism of pain and injury formation. Muscle pain and injury occurred in precompetition training, especially in freshmen. After heavy load, muscle soreness occurred, causing DOMS and developing into muscle injury. Affected by the external climate environment, sudden muscle soreness and injury are a gradual transformation process with DOMS as the boundary, which is the comprehensive result of exercise load, water, energy, and material metabolism; control load intensity, water supplement, and energy and material supplement can effectively prevent the occurrence of DOMS, and timely recovery after DOMS symptoms can effectively avoid the occurrence of sports injury. According to the different intensity of exercise, it is of great significance to clarify the mechanism of DOMS and explore effective prevention methods for physical education and sports training.

## 1. Introduction

As a continuation of physical education, the school sports meeting has an important reference value for testing students' physical quality, sports ability, and physical education level. The precompetition training of freshmen after entering school in autumn is a concentrated period of sports muscle pain and injury. The sports meeting of Guangxi University of science and technology is held at the beginning of November every year, which is representative in time and nature. It is similar to the sports meeting of most universities in Guangxi. The research on muscle pain and injury in precompetition training is of sample significance to other universities. In the precompetition training, a large number of students have muscle ache, *delayed onset muscle soreness* (DOMS) and other symptoms, and even muscle injury, especially a large number of freshmen show more obvious; the body finds it difficult to recover to participate in the school sports meeting; some of them have left old injuries and even have not fully recovered after sophomore year. Freshmen have just left high school and entered college. They are eager to get excellent results, have not dealt with the experience of increasing sports load, have ignored the sports health problems, and have become a group prone to exercise-induced muscle pain and injury. The occurrence of injuries has a negative impact on students' learning, life, and physical and mental health, as well as the development of physical education and sports training, weakening the enthusiasm of injured students to participate in sports in the future. The related literature lacks internal mechanism research on this special period, combined with the climate characteristics and the discomfort caused by a large number of freshmen participating in sports training. It is of great significance to analyze various factors that lead to muscle pain and injury and to study the internal mechanism of pain, so as to find an effective way to deal with muscle pain and prevent DOMS and muscle injury and serve school physical education.

## 2. Methodology

In the field of track and field, 125 students who participated in the prematch training of the school sports meeting were randomly selected as the research objects.

By means of interview, on-site observation, and mathematical statistics, the data of muscle pain and injury in the process of athletes' training were obtained, the data were consulted, and the internal mechanism of muscle pain and injury was studied based on the mechanism of DOMS. The injury type, muscle pain type, pain degree, exercise ability, and recovery time were analyzed.

## 3. Results and Discussion

### 3.1. Sports and Pain and Injury

The part of muscle pain in sports training is related to the muscle groups used in work. In the running events, the proportion of ache in middle and long distance running is lower than that in sprint, and the incidence of DOMS and injury is also lower than that in sprint. The incidence of ache, DOMS, and injury in jumping events is higher, and the incidence of ache, DOMS, and injury in middle and third-level jumping events is 100%, and the injury rate is 87.5%. The incidence of ache, DOMS, and injury in throwing events is 100%. The incidence of soreness, DOMS, and injury was the highest compared with other groups. It can be seen from Table 1 that the total number of people with pain is 101, accounting for 80.8% of the total, the number of people with DOMS is 91, accounting for 72.8% of the total, the total number of people with injury is 65, and the total injury rate is 52%. DOMS is between pain and injury. Sudden muscle soreness can be recovered in a short period of time and generally will not cause sports injury. If the recovery is unfavorable, a large part of it will be converted into DOMS, which will lead to injury. DOMS has a high correlation with muscle injury and the intensity of exercise load. With the increase of exercise intensity, the incidence of muscle soreness and muscle injury increases gradually. Although aerobic exercise has a large load, such as middle and long distance running, the incidence of DOMS is low; the incidence of DOMS in throwing and jumping events with a large load intensity is high, which is very easy to cause muscle injury. It is very important to study the mechanism of the generation, development, and disappearance of DOMS.

### 3.2. Discussion on the Mechanism of DOMS

DOMS refers to the feeling of muscle pain or discomfort after engaging in the unaccustomed exercise. The degree of discomfort occurs in the first 24 hours after exercise, reaches the peak in 24–72 hours, and then gradually relieves and disappears in about 5–7 days [1]. Since Hough discovered the phenomenon of DOMS in 1902, there is no unified explanation for the mechanism of DOMS at home and abroad. At present, there are mainly representative theories such as *lactic acid theory*, *muscle spasm theory, injury theory, inflammation theory,* and *enzyme escape theory* [2], but the above single theories cannot clearly explain the real cause of DOMS, and the prevention and control measures for DOMS cannot really work. Therefore, it is necessary to sort out and summarize the existing research results and explore the path of DOMS production, combined with various influencing factors. This paper mainly focuses on the metabolism of substance and energy, from the macrosystem integration effect to the microcombination of transverse bridge and actin in the theory of myofilament gliding, in order to provide a new way to clarify the mechanism of DOMS.

#### 3.2.1. Exercise and Lactate

The work of has shown that lactate produced by exercise is not the cause of DOMS; the works of show that the energy consumption, oxygen consumption, and lactic acid produced by muscle centrifugal contraction were less than that of centripetal contraction, but the DOMS produced was more serious. For example, the incidence of DOMS was 100% when the legs of the first and second jumps of the third jump landed in the ground. Lactate may cause fatigue related muscle pain, but it cannot be explained that lactate produced during exercise can cause delayed pain after 24–48 hours [3]. It can be seen that the production of lactic acid in muscle during exercise may lead to two different pain results: muscle soreness and DOMS. There are some similarities between the two mechanisms and pathways, but there are obvious differences. There are two main ways of glucose metabolism in human body: aerobic oxidation (under aerobic condition) and glycolysis (under anaerobic condition); the tricarboxylic acid cycle is the common way for sugar, fat, and protein to decompose in vivo. Under certain conditions, the three major energy substances take the tricarboxylic acid cycle as the hub and pyruvate, acetylcoa, etc., as the intersection point for mutual transformation [4].

During strenuous exercise, the muscle lacks oxygen supply, which produces lactic acid through glycolysis and releases energy for ATP resynthesis; due to the lack of enzyme in muscle that reversely transforms into glucose, the lactic acid in the muscle can no longer be converted into glycogen; when the oxygen supply is sufficient, most of the lactic acid can be oxygenated into CO_2_, H_2_O, and energy; about 17–25% of the lactic acid diffuses into the blood, and regenerate glycogen or glucose in the liver by gluconeogenesis, which is called lactate cycle, can avoid the loss of fuel and the accumulation of muscle lactate, leading to early muscle fatigue or acidosis [5]. During short-time vigorous exercise, energy consumption mainly depends on glycolysis.

The process of lactate production cannot explain DOMS alone, so it is necessary to combine with lactate removal pathway. Lactic acid produced by glycolysis can be removed mainly through three ways, as shown in Figure 1, and a small part can be directly removed from the body with urine and sweat. Under the action of lactate dehydrogenase, lactate is transformed into pyruvate when oxygen supply is sufficient and then enters mitochondria to generate AcCoA, which is oxidized to CO_2_, H_2_O, and energy through the tricarboxylic acid cycle.

#### 3.2.2. The Relationship between Lactic Acid and DOMS

When the body participates in the exercise without O_2_, there are two situations: one is that the exercise load is light and a small amount of lactate is produced, but the body has adapted to achieve the dynamic balance of production and decomposition so that the internal environment of lactate is kept at a low concentration level; the other is that the body cannot adapt to the increase of exercise load, and the large amount of lactic acid produced in an instant cannot be decomposed or removed in a short time, large amount of lactate cannot be decomposed or removed in a short time, and the dynamic balance between production and decomposition is broken, resulting in the accumulation of lactate. The hydrolysis and synthesis of ATP consume a lot of O_2_ and energy. Energy materials such as glycogen are mainly supplied by glycolysis: ADP + CP + energy is used to synthesize ATP + C, which produces amount of CO_2_ and metabolites (including lactic acid). CO_2_ + H_2_O = H_2_CO_3_ makes the internal environment acidified more seriously. With the increase of exercise load, fat, and protein gradually participating in energy supply, producing acid phosphates, ammonium salts, and other substances and making the internal environment of muscle tissue lose its steady state and pH drop, the inherent acid-base balance is broken, temperature rise makes the activity of enzyme decrease, leading to metabolic disorder, ATP energy supply is blocked, energy loss cannot be supplemented in time, and metabolic product removal is blocked, there is muscle tissue ache, and the work ability drops. The receptors of nerve endings in muscle tissue continue to produce local inflammation and induce DOMS under the joint action of physical stimulation (mechanical strain and temperature rise) and chemical stimulation (internal environment acidification) generated by movement; DOMS cannot be eliminated before the inflammation disappears. Lactic acid accumulation changes the internal environment, hinders the patency of energy supply, and increases the local body temperature, but it is not the direct cause of DOMS.

#### 3.2.3. Energy Supply System and Lactate and DOMS

The relationship between different exercise loads and lactate and DOMS was discussed from three energy supply systems. Because lactate cannot explain DOMS alone, in addition to the production of lactate by *glycolysis*, the *phosphagen system* and the *aerobic system* were investigated. The working principle of muscle tissue confirms the increasing exercise load until the submaximum (such as marathon) due to the sufficient O_2_ supply; glycogen decomposes completely without lactic acid accumulation and DOMS phenomenon, so the accumulation of lactic acid is related to the sudden increase of exercise load, which is beyond the adaptive range of the body. A large number of experiments have proved that DOMS can be produced by intensive exercise in a short period of 1-2 minutes, such as pull-up and sit ups, which are mainly powered by *glycolysis* and *phosphagen system*. DOMS has a significant common feature, which is the decrease of ATP synthesis efficiency and the change of substance metabolism in cells [6]. Therefore, we focus on *phosphagen system*, which mainly provides energy for the fast maximum power, namely, explosive power, in the first 10 seconds or so of exercise.

### 3.3. Inference of the Relationship between Muscle Pain, DOMS, and Injury Degree

The injury degree of muscle tissue is directly proportional to the recovery time and inversely proportional to the exercise ability. The more serious the injury degree is, the longer the recovery time is and the weaker the exercise ability is. The injury degree of DOMS can be indirectly inferred. Experiments show that, in addition to DOMS produced by high-intensity centrifugal exercise, there will be a drop in muscle strength immediately after exercise [7], and a decrease in the range of joint activity lasting for 1–4 days, and then, it gradually recovers [8]. From Table 2, it can be seen that the injury degree of DOMS is between muscle pain and muscle strain. The part of muscle pain was unapparent and the part of DOMS was concentrated in the whole muscle, but the pain focus was not obvious, and the pain focus of muscle injury was obvious. DOMS is a delayed subjective discomfort, involving the consumption of material and energy.

### 3.4. DOMS Threshold Theory

The excitation and contraction of muscle tissue come from the action potential of muscle fibers. The origin of DOMS is also from the action potential of motor unit, so it has the similar characteristics of action potential *full or none*, *nonattenuation conduction,* and *pulse type* [4]. It is impossible to produce DOMS as soon as exercise is performed. The stimulation intensity of individual DOMS is called “individual DOMS threshold,” and different individuals have great differences. Once any stimulus reaches the threshold value of individual DOMS, DOMS will be produced and reach the maximum value. The pain level will not be changed by the stimulus, and then, it gradually subsides to complete the whole process of DOMS. This explains that once DOMS is produced, it cannot be interrupted or stopped immediately, and various sports and treatment recovery methods are difficult to work. Exercise does not affect the natural recovery of DOMS, and the exercise induced by DOMS will not cause the accumulation of DOMS symptoms [9]. Once DOMS is generated, it will spread to the whole muscle participating in the movement, and the pain will not be weakened due to the increase of the transmission distance, which explains that the whole muscle tissue produces the same pain, and the focus of the pain is unapparent.

In a period of time, after the recovery of DOMS, the same load no longer causes DOMS, which explains that two consecutive DOMS have time intervals that should not be present. Continuous centrifugal exercise with repetition no more than the first training load will neither affect the recovery process of DOMS produced by the first training nor aggravate the muscle damage. However, the rest interval is too long (it varies from person to person, and the experiment proves that it is about 15–30 days). The same load can cause DOMS, and the adaptation time of the load obtained by the body disappears.

## 4. Conclusion

It is of great practical significance to teach the basic knowledge of exercise physiology and to let students master the scientific exercise methods for improving the students' health level and physical quality and promoting the development of physical education. The freshmen's lack of experience to participate in high-intensity training, strengthens sports health education and popularizes scientific exercise methods and prevention measures of general sports pain and injury. Especially for high jump, long jump, javelin, shot put, and other fast strength events [10], it is easy to cause muscle soreness symptoms and even injury. In training, we should arrange exercise load reasonably; especially, the increase of exercise intensity has a gradual process, masters the matching of exercise amount and intensity, and pays attention to the recovery of physical fitness.

Under the dry and hot climate in South China in autumn, the water consumption of the body is accelerated, which is easy to cause the body to lose water. In the process of training, according to the principle of a small amount and many times, we should supplement water for the body and keep the internal environment relatively in a stable state, which is conducive to the material exchange between muscle tissues and cells and the timely elimination of metabolites. Supplement energy maintains the normal operation of the energy supply system of the body, pays attention to nutrition diet before and after training, and maintains the nitrogen balance of the body and the activity of various enzymes. When inorganic salt was added, Ca^2 +^ which triggered action potential was added in time and Na^+^ and K^+^ were added to maintain the excitability of nerve impulse of muscle cells.

The development of muscle injury from DOMS is a process of increasing pain and body load. Therefore, we should pay attention to the active recovery of body fatigue and sudden muscle ache. After DOMS occurs, we should take rest for some time and reduce the exercise during the period when the pain reaches the maximum value, so as to avoid the aggravation of pain and tissue damage and develop into muscle damage. Preventing DOMS and taking timely rest measures after DOMS symptoms, we can effectively avoid the occurrence of sports muscle injury, enable students to learn the general knowledge of self judgment of muscle soreness symptoms and self-protection, and provide theoretical reference for other school sports meeting training and competition to prevent sports muscle pain and injury.

## Figures and Tables

**Figure 1:** Glycolysis process.

**Table 1:** Sports events and pain and injury analysis.

Project (people number)	Run (61)	Jump (24)	Throw(40)
	Distance race (25) and sprint (36)	High jump (6), broad jump (10), and triple jump (8)	Shot put (12), back throw solid ball (16), and softball throw (12)
Pain of body parts	Quadriceps, gluteus, gastrocnemius, and biceps	Quadriceps, gluteus, gastrocnemius, psoas, dorsal, and abdominal	Deltoid, erector, dorsal, abdominal, triceps brachii, quadriceps femoris, and medial thigh
Ache people number (%)	16 (64) 30 (83.3)	5 (83.3) 8 (80) 8 (100)	10 (83.3) 16 (100) 12 (100)
DOMS people number (%)	12 (48) 24 (66.7)	5 (83.3) 7 (70) 8 (100)	9 (75) 14 (87.5) 12 (100)
Injure people number (%)	4 (16) 20 (55.6)	3 (50) 6 (60) 7 (87.5)	8 (66.7) 6 (37.5) 11 (91.7)
Project injury rate (%)	19.2	12.8	20

**Table 2:** Recovery of muscle pain and injury.

Injury types	Recovery time	Ability to exercise	Pain focus
Muscle soreness	Recover in hours	Ability decline	Unapparent
DOMS	5–7 days	Dyskinesia	More concentrated
Muscle injury	About a month	Unable to exercise	Focus on one place

## Data Availability

The datasets used and/or analyzed during the current study are available from the corresponding author upon reasonable request.

## References

[1] Clarkson P. M., Nosaka K., Braun B. (1992). Muscle function after exercise-induced muscle damage and rapid adaptation. *Medicine & Science in Sports & Exercise*.

[2] Cheung K., Hume P., Maxwell L. (2003). Delayed onset muscle soreness: treatment strategies and performance factors. *Sports Medicine (Auckland, N.Z.)*.

[3] Xu J. (1993). A review on the mechanism of delayed onset muscle soreness. *Sport Science*.

[4] Wang R., Su Q. (2002). *Sports Physiology*.

[5] Wang B., Hua M. (1992). *Sports Physiology*.

[6] Brown S. J., Child R. B., Donnelly A. E., Saxton J. M., Day S. H. (1996). Changes intiuman skeletal muscle contractile function following stimulated eccentric exercise. *DurjApplphysi*.

[7] Wang X. (2015). *Study on the Effect of Moxibustion on DOMS After Exercise*.

[8] Serravite D. H., Perry A., Jacobs K. A., Adams J. A., Harriell K., Signorile J. F. (2014). Effect of whole-body periodic acceleration on exercise-induced muscle damage after eccentric exercise. *International Journal of Sports Physiology and Performance*.

[9] Chong Z. (2005). Development of the research on delayed onset muscle soreness. *Journal of Physical Education*.

[10] Tian M., Liu D. (2012). *Sports Training*.

